RETRACTED

# Grape Seed Proanthocyanidins Inhibit Melanoma Cell Invasiveness by Reduction of PGE_2_ Synthesis and Reversal of Epithelial-to-Mesenchymal Transition

**DOI:** 10.1371/journal.pone.0021539

**Published:** 2011-06-27

**Authors:** Mudit Vaid, Tripti Singh, Santosh K. Katiyar

**Affiliations:** 1 Department of Dermatology, University of Alabama at Birmingham, Birmingham, Alabama, United States of America; 2 Comprehensive Cancer Center, University of Alabama at Birmingham, Birmingham, Alabama, United States of America; 3 Birmingham VA Medical Center, Birmingham, Alabama, United States of America; University of Pennsylvania School of Medicine, United States of America

## Abstract

Melanoma is the leading cause of death from skin disease due, in large part, to its propensity to metastasize. We have examined the effect of grape seed proanthocyanidins (GSPs) on melanoma cancer cell migration and the molecular mechanisms underlying these effects using highly metastasis-specific human melanoma cell lines, A375 and Hs294t. Using *in vitro* cell invasion assays, we observed that treatment of A375 and Hs294t cells with GSPs resulted in a concentration-dependent inhibition of invasion or cell migration of these cells, which was associated with a reduction in the levels of cyclooxygenase (COX)-2 expression and prostaglandin (PG) E_2_ production. Treatment of cells with celecoxib, a COX-2 inhibitor, or transient transfection of melanoma cells with COX-2 small interfering RNA, also inhibited melanoma cell migration. Treatment of cells with 12-O-tetradecanoylphorbol-13-acetate, an inducer of COX-2, enhanced the phosphorylation of ERK1/2, a protein of mitogen-activated protein kinase family, and subsequently cell migration whereas both GSPs and celecoxib significantly inhibited 12-O-tetradecanoylphorbol-13-acetate -promoted cell migration as well as phosphorylation of ERK1/2. Treatment of cells with UO126, an inhibitor of MEK, also inhibited the migration of melanoma cells. Further, GSPs inhibited the activation of NF-κB/p65, an upstream regulator of COX-2, in melanoma cells, and treatment of cells with caffeic acid phenethyl ester, an inhibitor of NF-κB, also inhibited cell migration. Additionally, inhibition of melanoma cell migration by GSPs was associated with reversal of epithelial-mesenchymal transition process, which resulted in an increase in the levels of epithelial biomarkers (E-cadherin and cytokeratins) while loss of mesenchymal biomarkers (vimentin, fibronectin and N-cadherin) in melanoma cells. Together, these results indicate that GSPs have the ability to inhibit melanoma cell invasion/migration by targeting the endogenous expression of COX-2 and reversing the process of epithelial-to-mesenchymal transition.

RETRACTED

## Introduction

Melanoma is the leading cause of death from skin disease due to its propensity to metastasis [1], [2], and is increasing rapidly in children [3]. Although, melanoma is less common than other types of skin cancers, it causes the majority (75%) of skin cancer-related deaths [1], [4]. The American Cancer Society estimated that in 2008, there were 8,420 melanoma-associated deaths in the U.S. and the number of new cases of invasive melanoma was estimated at 62,480 [1]. Solar ultraviolet (UV) radiation is a recognized risk factor for the development of skin cancers, including melanoma. Exposure of the skin to UV radiation induces an increase in the expression levels of cyclooxygenase -2 (COX-2), a rate-limiting enzyme that catalyzes the conversion of arachidonic acid to prostaglandins (PGs) [5], [6]. These inflammatory mediators have been identified as a risk factor for the development of skin cancers [5], [6], and thought to play a central role in orchestrating the multiple events involved in cancer invasion and metastasis [7], [8]. Since, melanoma is a highly malignant cancer with a potent capacity to metastasize distantly, an approach that decreases its metastatic or invasive ability may facilitate the development of an effective strategy for its treatment or prevention.

Dietary phytochemicals offer promising new options for the development of more effective strategies for the prevention of cancer cell invasion, migration, or metastasis, and thus can be utilized as complementary and alternative medicine. Grape seed proanthocyanidins (GSPs) are promising phytochemicals that have shown anti-carcinogenic effects in some murine models and exhibit no apparent toxicity *in vivo* [9]–[11]. GSPs contain primarily proanthocyanidins (89%), which constitute dimers, trimers, tetramers, and oligomers of monomeric catechins and/or (-)-epicatechins, as described previously [10]. They are readily available as an extract of grape seeds and this extract, rather than the individual constituents, has been examined as an anti-carcinogenic agent against some forms of cancers [9]. It is believed that at least some of the constituents present in the extract may act synergistically and thus this product can be more effective than any single constituent. GSPs have been shown to inhibit UV radiation-induced skin cancer in mouse model [10] but its chemopreventive effect on the migration or invasive potential of melanoma cancer cells has not been explored.

In this study, we assessed the chemotherapeutic effects of GSPs on the migration potential of human melanoma cells, as the migration of cancer cells is a major event in the metastatic cascade. For this purpose, two highly metastasis-specific melanoma cancer cell lines were selected: one is A375 which is *BRAF* mutated and activating mutations of the protooncogene *BRAF* have been observed in approximately 50% of malignant melanomas. Second cell line is Hs294t, which is also highly metastatic but not *BRAF* mutated. In this study, we characterized the role of COX-2 and its metabolite PGE_2_ on the migration of human melanoma cancer cells and ascertained whether GSPs have any suppressive effects on the COX-2-mediated migration of these cells. Epithelial-to-mesenchymal transition (EMT), the process whereby epithelial cells transform into mesenchymal cells, has recently been shown to be relevant for cancer and cancer metastasis. During EMT, cancer cells lose expression of proteins that promote cell-cell contact such as E-cadherin and acquire mesenchymal markers such as vimentin, fibronectin and N-cadherin, which promote cell invasion and metastasis [12]. The EMT has also been associated with higher levels of inflammation or inflammatory mediators, and therefore we have also checked whether inhibition of COX-2 expression by GSPs in melanoma cells is associated with reversal of EMT and that leads to inhibitory effect on melanoma cell migration. Here, we present evidence that GSPs inhibit the invasiveness or migratory behavior of melanoma cancer cells through inhibition or reversal of EMT in melanoma cells and that GSPs do so through a process that involves the reduction in COX-2 expression and PGE_2_ production.

RETRACTED

## Materials and Methods

### Source and composition of GSPs

GSPs were received from Kikkoman Corporation (Noda, Japan). Quality control of GSPs is maintained by the company on lot-to-lot basis. GSPs contain approximately 89% proanthocyanidins, with dimers (6.6%), trimers (5.0%), tetramers (2.9%) and oligomers (74.8%), as described earlier [10], [11], and are stable for at least two years when refrigerated at 4°C.

### Cell lines and cell culture conditions

The human melanoma cells lines, A375 and Hs294, were purchased from the American Type Culture Collection (Manassas, VA). The cell lines were cultured as monolayers in RPMI 1640 culture medium supplemented with 10% heat-inactivated fetal bovine serum (Hyclone, Logan, UT), 100 µg/ml penicillin, and 100 µg/ml streptomycin and maintained in an incubator with 5% CO_2_ at 37°C. The GSPs were dissolved in a small amount of dimethylsulfoxide (DMSO), which was added to the complete cell culture medium [maximum concentration of DMSO, 0.1% (v/v) in media] prior to addition to sub-confluent cells (60–70% confluent). Cells treated with DMSO only served as a vehicle control. Normal human epidermal melanocytes (HEMa-LP, Cat. No. C-024-5C) were commercially obtained from Invitrogen (Carlsbad, CA), and were cultured in HMGS-2 medium supplemented with human melanocyte growth supplement provided by the supplier. To determine the effect of GSPs on 12-O-tetradecanoylphorbol-13-acetate (TPA)- or PGE_2_-mediated effects, GSPs were added in cell culture medium at least 30 minutes before the treatment of the cells with TPA, PGE_2_ or any other agent.

RETRACTED

### Antibodies, chemicals and reagents

Antibodies specific for COX-2 and an enzyme immunoassay kit for PGE_2_ analysis were obtained from Cayman Chemicals (Ann Arbor, MI). Celecoxib, PGE_2_ and 12-O-tetradecanoylphorbol-13-acetate (TPA) were purchased from Sigma Chemical Co. (St. Louis, MO). Boyden Chambers and polycarbonate membranes (8 µm pore size) for cell migration assays were obtained from Neuroprobe, Inc. (Gaithersburg, MD). The antibodies specific to N-cadherin, keratin-8, -18 and fibronectin were obtained from Santa Cruz Biotechnology (Santa Cruz, CA), while antibodies for vimentin, E-cadherin, NF-κB, IKKα and IκBα were purchased from Cell Signaling Technology (Beverly, MA) while desmoglein-2 was obtained from Abcam (Cambridge, MA). The secondary antibodies conjugated with Alexa Fluor 488 or Alexa Fluor 594 were purchased from Invitrogen (Carlsbad, CA).

### Cell migration or invasion assay

The migration capacity of melanoma cancer cells was determined *in vitro* using Boyden Chambers (Gaithersburg, MD) in which the two chambers were separated with matrigel coated Millipore membranes (6.5 mm diameter filters, 8 µM pore size), as detailed previously [13]. Briefly, melanoma cells (1.5×10^4^ cells/100 µL serum-reduced medium) were placed in the upper chamber of Boyden chambers, test agents were added alone, or in combination, to the upper (200 µL) chamber, and the lower chamber contained the medium alone (150 µL). Chambers were assembled and kept in an incubator for 24 h. After incubation, cells from the upper surface of Millipore membranes were removed with gentle swabbing and the migrant cells on the lower surface of membranes were fixed and stained with either hematoxylin or crystal violet. Membranes were then washed with distilled water and mounted onto glass slides. The membranes were examined microscopically and cellular migration was determined by counting the number of stained cells on membranes in at least 4–5 randomly selected fields using an Olympus BX41 microscope. Representative photomicrographs were obtained using a Qcolor5 digital camera system fitted to an Olympus BX41 microscope. Each cell migration experiment was repeated at least three times.

RETRACTED

### PGE_2_ immunoassay for quantitation of prostaglandin E2

The analysis of PGE_2_ in cell homogenates was performed using the Cayman PGE_2_ Enzyme Immunoassay Kit (Ann Arbor, MI) following the manufacturer's instructions. Briefly, at indicated time points, cells were harvested and homogenized in 100 mM phosphate buffer, pH 7.4 containing 1 mM ethylenediamine tetraacetic acid and 10 µM indomethacin using a homogenizer. Homogenates were centrifuged and the supernatants were collected and analyzed for PGE_2_ concentration according to the manufacturer's instructions.

### COX-2-siRNA transfection of A375 and Hs294t cells

Human-specific COX-2 siRNA was transfected into A375 and Hs294t cells using the siRNA Transfection Reagent Kit (Santa Cruz Biotechnology, Inc.; Santa Cruz, CA) according to the manufacturer's protocol. Briefly, 2×10^5^ cells/well were seeded in a 6-well plate and allowed to grow to 70% confluency. The COX-2 siRNA mix with transfection reagents was overlaid on the cells for approximately 6 h at 37°C and transferred into 2× growth medium for about 18–20 h. At 24 h post-transfection, fresh medium was added to the cells and the cells were incubated for an additional 48 h. Thereafter, cells were harvested and subjected to the cell migration assay. The knockdown of COX-2 expression in cells after transfection was confirmed using western blot analysis.

### NF-κB/p65 activity assay

For quantitative analysis of NF-κB/p65 activity, the NF-κB Trans^AM^ Activity Assay Kit (Active Motif, Carlsbad, CA) was used following the manufacturer's protocol. For this purpose, the nuclear extracts of cells were prepared using the Nuclear Extraction Kit (Active Motif, Carlsbad, CA) following the manufacturer's instructions, and as performed previously [14]. Absorbance was recorded at 450 nm using absorbance at 650 nm as the reference. The results are expressed as the percentage of the optical density of the non-GSPs-treated control group.

### Preparation of cell lysates and western blot analysis

Following treatment of melanoma cells for the indicated time periods with or without GSPs or any other agent, the cells were harvested, washed with cold PBS and lysed with ice-cold lysis buffer supplemented with protease inhibitors, as detailed previously [15]. Equal amounts of proteins were resolved on 10% Tris-Glycine gels and transferred onto a nitrocellulose membrane. After blocking the non-specific binding sites, the membrane was incubated with the primary antibody at 4°C overnight. The membrane was then incubated with the appropriate peroxidase-conjugated secondary antibody and the immunoreactive bands were visualized using the enhanced chemiluminescence reagents. To verify equal protein loading, the membrane was stripped and reprobed with anti-β actin antibody.

RETRACTED

### Immunofluorescent detection of EMT biomarkers in cells

In order to determine whether GSPs inhibit cell migration of melanoma cells is associated with reversal of epithelial-to-mesenchymal transition, the A375 melanoma cells were either treated with various concentrations of GSPs or celecoxib or TPA for 24 h. After 24 h, cells were harvested and cell lysates were prepared for western blotting for the analysis of epithelial and mesenchymal biomarkers. Cells were also used for cytostaining for the detection of EMT biomarkers such as vimentin, fibronectin and N-cadherin. Briefly, after harvesting the cells, cells were processed for cytospin (1×10^5^ cells/slide). Cells were fixed with chilled methanol at −20°C for 10 minutes and non specific binding sites were blocked with 2% bovine serum albumin (Sigma, St. Louis, MO) in PBS for 30 min. Cells were then incubated with antibodies specific to EMT biomarkers for 2 h at room temperature. The cells were washed with PBS and antigen was detected by an Alexa Fluor-conjugated secondary antibody. Goat anti-rabbit IgG labeled with green-fluorescent Alexa Fluor 488 dye was used for detection of N-cadherin and vimentin, while donkey anti-mouse IgG labeled with red-fluorescent Alexa Fluor 594 was used for the detection of the expression of desmoglein 2. Cells were finally mounted with Vectashield mounting medium for fluorescence with DAPI (Vector Laboratories, Burlingame, CA) before they were observed under fluorescence microscope and photographed.

### Statistical analysis

For migration assays, the control and GSPs-, TPA- or PGE_2_-treatment groups or combined-treatment groups separately were compared using one-way analysis of variance (ANOVA) followed by *post hoc* Dunn's test using GraphPad Prism version 4.00 for Windows, GraphPad Software, San Diego, California, USA, www.graphpad.com. All quantitative data for cell migration are shown as mean ± SD/microscopic field. In each case *P*<0.05 was considered statistically significant.

## Results

### Comparative invasiveness of human melanoma cells and normal human epidermal melanocytes

First, we examined the migration capacity of melanoma cells and compared this capacity with normal human epidermal melanocytes under identical conditions. For this purpose, cells were incubated in Boyden chambers for 24 h to assess their migration capability. As shown in Figure 1A, the cell migration capacity of melanoma cells was significantly higher (*P*<0.001) than normal human epidermal melanocytes. The migration of A375 cells, which are *BRAF* mutated, was greater (390±14 cells/microscopic field) than Hs294t cells (340±12 cells/microscopic field), which are metastasis-specific but not *BRAF*-mutated. Under identical conditions, migration of normal human epidermal melanocytes was lower (19±4 cells/microscopic field) than melanoma cells.

RETRACTED

**Figure 1:** Effect of GSPs on melanoma cell migration. (**A**) Migration ability of human melanoma cells and comparison with normal human epidermal melanocytes (HEMa). Equal numbers of human melanoma cells (A375 and Hs294t) and HEMa were subjected to cell migration using standard Boyden chamber assay. Twenty four h later, migratory cells were detected on the membrane after staining with crystal violet. The migratory cells were counted and the results expressed as the mean number of migratory cells ± SD per microscopic field (n = 3). Significantly lower *versus* melanoma cells, ^*^ *P*<0.001. (**B**) Treatment of human melanoma cancer cells (A375 and Hs294t) with GSPs for 24 h inhibit migration of cells in a concentration-dependent manner compared to non-GSPs-treated control cells. (**C**) The migratory cells were counted and the results expressed as the mean number of migratory cells ± SD/microscopic field. Significant inhibition *versus* non-GSPs-treated control, ^*^ *P*<0.001.

### GSPs inhibit human melanoma cancer cell migration

We determined whether treatment of A375 and Hs294t human melanoma cells with GSPs inhibited their invasiveness or migration using Boyden chamber cell migration assays. First, screening experiments were performed to determine the effects of lower concentrations of GSPs (µg/mL). The selection of the concentrations of GSPs was based on consideration of their relevance and achievability *in vivo*. As shown in Figure 1B, relative to untreated control cells, treatment of cells with GSPs at concentrations of 0, 10, 20 and 40 µg/mL reduced the invasive potential of A375 and Hs294t cells in a concentration-dependent manner. The density of the migrating cells on the membrane after staining with crystal violet is shown in Figure 1B, and the numbers of migrating cells/microscopic field are summarized in Figure 1C. The cell migration was inhibited by 22 to 64% (*P*<0.01−0.001) in A375 cells and by 29–69% (*P*<0.01−0.001) in Hs294t cells in a concentration-dependent manner after treatment with GSPs for 24 h. A similar but comparatively higher inhibitory effect on cell migration was observed at the 48 h time point (data not shown). To confirm that the inhibition of cancer cell migration by GSPs was a direct effect on migration ability, and that was not due to a reduction in cell viability, a trypan blue assay was performed using cells that were treated identically to those used in the migration assays. Treatment of A375 and Hs294t cells with various concentrations of GSPs (0, 10, 20 and 40 µg/mL) for 24 h had no significant effect on cell viability or cell death (data not shown).

RETRACTED

### The inhibitory effect of GSPs on invasiveness of melanoma cells is associated with the reduction of endogenous COX-2 expression and reduction of PGE_2_ synthesis

To determine whether the inhibitory effect of GSPs on the migration of the melanoma cells is associated with inhibition of endogenous COX-2 expression, we determined the levels of COX-2 in lysates of cells from the various treatment groups using western blot analysis. As shown in Figure 2A, treatment of A375 and Hs294t cells with GSPs reduced the levels of COX-2 expression in a concentration-dependent manner as compared to the expression in untreated controls. As the COX-2 metabolite, PGE_2_, has been implicated in COX-2-mediated effects including cancer cell metastasis; we determined the levels of PGE_2_ in the GSPs-treated cells. Our results revealed that treatment with GSPs for 24 h resulted in significant reduction in the production or synthesis of PGE_2_ in both A375 (19–76%, *P*<0.001) and Hs294t (18–71%, *P*<0.001) cells in a concentration-dependent manner (Figure 2B), suggesting that GSPs-induced reduction in PGE_2_ production is associated with an inhibitory effect of the GSPs on COX-2 expression and inhibition of cell migration in these cells.

**Figure 2:** Effect of GSPs on COX-2 expression, PGE_2_ production and cell migration in melanoma cells. (**A**) Effect of GSPs on the endogenous basal level of COX-2 in A375 and Hs294t cells. The levels of COX-2 were determined in cell lysates using western blot analysis. (**B**) Dose-dependent effect of GSPs on the levels of PGE_2_ in melanoma cells. The levels of PGE_2_ are expressed in terms of pg/mg protein± SD, n = 3 independent experiments. Significant inhibition of PGE_2_ level by GSPs *versus* non-GSPs-treated controls, ^*^ *P*<0.001. (**C**) Down-regulation of endogenous COX-2 reduces melanoma cell migration. Treatment of A375 and Hs294t cells with celecoxib, a COX-2 inhibitor, inhibits cell migration in a dose-dependent manner. Significant difference *versus* control (non-celecoxib-treated) cells, ^¶^ *P*<0.05, ^*^ *P*<0.001. (**D**) Transfection of cells, both A375 and Hs294t, with COX-2 siRNA significantly decreases cell migration. A375 and Hs294t cells were transfected with COX-2 siRNA to knockdown COX-2 expression. Significant reduction of cell migration *versus* control siRNA-treated cells: ^*^ *P*<0.001. (**E**) Treatment of A375 and Hs294t cells with GSPs (20 and 40 µg/mL) inhibits PGE_2_-enhanced cell migration. The data on cell migration are summarized as a mean number of migratory cells ±SD/microscopic field. In each case, the migrating cells were counted at 4–5 different microscopic fields, and data are expressed as the mean number of migratory cells± SD/microscopic field, n = 3.

RETRACTED

### Selective COX-2 inhibitor inhibits melanoma cell migration

This experiment was performed to determine whether the inhibitory effect of GSPs on melanoma cell migration is mediated through its inhibitory effect on COX-2 expression. For this purpose, equal numbers of A375 and Hs294t cells were subjected to the cell migration assay after treatment with various concentrations of celecoxib (0, 5, 10, 20 µM), a well known inhibitor of COX-2, for 24 h. As shown in Figure 2C, treatment of the cells with celecoxib resulted in a dose-dependent reduction in the cell migration capacity of melanoma cells as compared with non-celecoxib-treated controls (*P*<0.05−0.001). These data suggested that the inhibition of constitutive levels of COX-2 expression is associated with the inhibition of melanoma cell migration.

### siRNA knock-down of COX-2 leads to reduction of melanoma cell migration

We further verified the role of COX-2 in cell migration through siRNA knock-down of COX-2 in the melanoma cells and examined whether it would lead to the inhibition of the cell migration in these cells. The transfection of A375 and Hs294t cells with COX-2 siRNA resulted in significant reduction of cell migration in A375 (85%, *P*<0.001) and Hs294t (86%, *P*<0.001) cells after 24 h as compared to the migration of control siRNA-transfected A375 and Hs294t cells (Figure 2D).

### GSPs inhibit PGE_2_-induced cell migration of melanoma cells

As the effects of COX-2 are mediated through its metabolites, such as PGE_2_, we examined whether GSPs inhibit PGE_2_-induced cell migration in human melanoma cells. For this purpose, A375 and Hs294t cells were treated with PGE_2_ (10 µM) with and without GSPs for 24 h and cell migration determined. We found that the treatment of melanoma cells with PGE_2_ resulted in a significant increase in cell migration (*P*<0.05) compared to the cells which were not treated with PGE_2_ (Figure 2E). Treatment of A375 and Hs294t cells with GSPs (20 or 40 µg/mL) resulted in a dose-dependent inhibition of PGE_2_ (10 µM)-induced cell migration (Figure 2E). As the inhibitory effect of GSPs on the migration of A375 and Hs294t cell lines was very similar, the subsequent studies were performed only with A375 cells.

### TPA, an inducer of COX-2, enhances melanoma cell migration, and GSPs inhibit TPA-induced cell migration

Treatment of skin with TPA stimulates the levels of COX-2 expression [11], [16]; therefore, the melanoma cells were treated with TPA for COX-2 stimulation, and thereafter determined the effect of TPA on the migration of melanoma cells. As shown in Figure 3A, treatment of A375 cells with TPA for 24 h resulted in significantly enhanced cell migration (*P*<0.01) compared to non-TPA-treated cells. To determine whether GSPs inhibit TPA-induced cell migration in human melanoma cells, A375 cells were treated with TPA (40 ng/mL) with and without the treatment of GSPs for 24 h. We found that the treatment of A375 cells with GSPs resulted in a dose-dependent inhibition of TPA-induced cell migration. A summary of the cell migration data for the various treatment groups is provided in Figure 3A. Treatment of cells with GSPs at the doses of 20 µg/mL and 40 µg/mL inhibited TPA-induced cell migration by 50% (*P*<0.01) and >100% (*P*<0.001) respectively.

RETRACTED

**Figure 3:** Effect of GSPs and celecoxib on TPA-induced activation of ERK1/2 and melanoma cell migration. (**A**) Effect of TPA or its combination with GSPs on melanoma cell migration. Treatment of A375 cells with TPA, a stimulator of COX-2, significantly enhances cell migration (**^†^** *P*<0.001) compared with non-TPA-treated control cells. (**B & C**) Treatment of A375 cells with TPA results in activation of ERK1/2. Treatment of cells with GSPs (40 µg/mL) or celecoxib (40 µM) inhibits TPA-induced activation of ERK1/2 protein, and simultaneously inhibits TPA-enhanced migration of melanoma cells. The data on cell migration capacity are summarized in Panel **C**. Significant inhibition versus TPA-treatment alone, ^*^ *P*<0.001. (**D**) Treatment of melanoma cells with MEK inhibitor (UO126, 80 µM) resulted in inhibition of the activation of ERK1/2 as well as inhibition of cell migration compared to non-MEK inhibitor-treated control cells. The data are expressed as the mean number of migratory cells± SD/microscopic field, n = 3. Significant difference versus controls ^*^ *P*<0.001.

### GSPs and celecoxib inhibit TPA-induced activation of ERK1/2 protein in melanoma cells

As activation of MAPK proteins has been implicated in the enhancement of COX-2 expression or an upstream regulator of COX-2, we examined the effect of TPA on activation of ERK1/2 in melanoma cells, and simultaneously checked the effect of GSPs or celecoxib on TPA-induced activation of ERK1/2. Western blot analysis revealed that treatment of A375 cells with TPA enhanced the activation of ERK1/2, however, treatment of cells with GSPs or celecoxib inhibited TPA-induced activation of ERK1/2, as shown in Figure 3B. We further checked the effect of GSPs and celecoxib on TPA-induced cell migration. Cell migration assay analysis revealed that both GSPs and celecoxib significantly inhibited TPA-induced cell migration of melanoma cells (Figure 3C). We further verified the role of activated ERK1/2 in melanoma cell migration by using the inhibitor of MEK (UO126). Cell migration assay revealed that treatment of A375 cells with UO126 significantly inhibited (*P*<0.001) melanoma cell migration (Figure 3D). A summary of data related with cell migration are also shown. Additionally, western blot analysis revealed that the level of activated ERK1/2 was also decreased after the treatment of cells with MEK inhibitor UO126, as shown in Figure 3D.

RETRACTED

### GSPs decrease the activation of NF-κB/p65 in melanoma cells: NF-κB is an important mediator of melanoma cell migration

COX-2 is a downstream target of NF-κB, therefore we assessed whether GSPs also affect the proteins of NF-κB family in melanoma cells. For this purpose, A375 cells were treated with various concentrations of GSPs (0, 10, 20 and 40 µg/mL) for 24 h, and thereafter cells were harvested and whole cell lysates and nuclear lysates were prepared. The results of western blot analysis revealed that treatment of cells with GSPs reduce the nuclear translocation of NF-κB/p65 in a dose-dependent manner (Figure 4A). The activity of NF-κB also was significantly reduced (25–70%, *P*<0.01 and *P*<0.001) after the treatment of cells with GSPs in a concentration-dependent manner (Figure 4B). The western blot analysis also revealed that treatment of GSPs resulted in the down-regulation of IKKα, an enzyme responsible for NF-κB activation, and degradation of IκBα (Figure 4A), which leads to the inactivation of NF-κB. To check whether NF-κB has a role in melanoma cell migration, A375 melanoma cells were treated with caffeic acid phenethyl ester (0, 5, 10 and 20 µg/mL), a potent inhibitor of NF-κB, and cell migration was determined. As shown in Figure 4C, treatment of cells with caffeic acid phenethyl ester resulted in a dose-dependent reduction of cell migration (24–78%) relative to untreated control cells, and it was similar to that observed on treatment of the cells with GSPs (Figure 1B).

**Figure 4:** Effect of GSPs on NF-κB activation. (**A**) Treatment of A375 cells with GSPs decreases the basal levels of NF-κB/p65 and IKKα while inhibiting the degradation of IκBα. After treatment of cells for 24 h with various concentrations of GSPs the cells were harvested and cytosolic and nuclear fractions were prepared and subjected to the analysis of NF-κB/p65, IKKα and IκBα using western blot analysis. Representative blot is shown from three independent experiments with identical results. (**B**) The activity of NF-κB/p65 in the nuclear fraction of cells after treatment with and without GSPs for 24 h was measured using NF-κB/p65-specific activity assay kit, n = 3. Activity of NF-κB/p65 is expressed in terms of percent of control (non-GSPs-treated) group. Significant decrease versus control: ^¶^ *P*<0.01, ^*^ *P*<0.001. (**C**) Treatment of A375 cells with caffeic acid phenethyl ester (CAPE), an inhibitor of NF-κB, for 24 h inhibits cell migration in a concentration-dependent manner. Data on cell migration capacity are summarized as the mean number of migratory cells ± SD/microscopic field, n = 3. Significant inhibition versus non-CAPE-treated cells: ^*^ *P*<0.001.

RETRACTED

### GSPs reverse epithelial-to-mesenchymal transition in melanoma cells

Activation of NF-κB has been implicated in inflammation-induced cancer development and progression, and has been identified as an important regulator of EMT in several cancer cell types [17]–[20]. As the inhibition of melanoma cell migration by GSPs is associated with the inactivation of NF-κB, we sought to determine whether GSPs also affect or reverse EMT in melanoma cells and that is responsible for their inhibitory effect on melanoma invasiveness. For this purpose, A375 cells were treated with GSPs for 24 h, and cell lysates were prepared for the western blot analyses of various epithelial and mesenchymal biomarkers. Our western blot analyses revealed that GSPs restored or increased the levels of the epithelial biomarkers, such as E-cadherin, keratin-18, keratin-8 and desmoglein 2 in melanoma cells compared to untreated controls. In contrast, the levels of mesenchymal biomarkers, such as N-cadherin, vimentin, fibronectin and SLUG, were reduced in melanoma cells after treatment with GSPs in a dose-dependent manner, as shown in Figure 5A. GSPs-induced changes or effects on these epithelial and mesenchymal biomarkers were also detected and analyzed using immunofluorescence staining (Figure 5B). Immunofluorescnce staining data revealed that treatment of A375 cells with GSPs for 24 h resulted in reduction of mesenchymal biomarkers, such as vimentin, fibronectin and N-cadherin which is evident by the intensity of staining of the cells. In contrast, GSPs enhanced the levels of epithelial biomarker, such as desmoglein 2, in melanoma cells which is evident by the strong intensity of fluorescence staining compared to untreated controls. Similar observations were also noted when cells were treated with celecoxib, a COX-2-specific inhibitor, in identical manner. Representative photomicrographs are shown from three independent experiments.

**Figure 5:** Treatment of melanoma cells with GSPs results in reversal of epithelial to mesenchymal transition. (**A**) Treatment of A375 cells with GSPs for 24 h enhances the levels of epithelial biomarkers in the cells, such as, the levels of E-cadherin, keratin-18, keratin-8 and desmoglein 2. Simultaneously the levels of mesenchymal biomarkers in melanoma cells, such as, vimentin, fibronectin, N-cadherin and SLUG were decreased dose-dependently. (**B**) Identification of the levels of epithelial and mesenchymal biomarkers in A375 cells after the treatment of cells with GSPs or celecoxib using immunocytostaining, as detailed in Materials and Methods. Treatment of A375 cells with GSPs (20 and 40 µg/mL) or celecoxib (20 µM) for 24 h resulted in reduced expression of vimentin, fibronectin and N-cadherine, while the level of desmoglein 2 was increased. Representative photomicrographs are representative of three independent experiments with similar results.

RETRACTED

### GSPs and celecoxib inhibit TPA-induced EMT biomarkers in melanoma cells

As TPA induces COX-2 expression as well as enhances cell migration in melanoma cells, we next examined whether TPA promotes EMT in melanoma cells and whether GSPs and celecoxib inhibit TPA-induced EMT in these cells. For this purpose, A375 melanoma cells were treated with either TPA or celecoxib alone or TPA with the treatment of GSPs for 24 h, cell lysates prepared and subjected to western blot analysis. As shown in Figure 6, TPA decreased the level of desmoglein 2 (an epithelial biomarker), while enhanced the levels of mesenchymal biomarkers (N-cadherin and vimentin) compared with untreated control cells. Celecoxib enhanced the level of desmoglein 2 while decreased the levels of N-cadherin and vimentin compared with untreated control melanoma cells. Further, as shown in Figure 6, GSPs increased or restore the level of desmoglein 2 in TPA-treated melanoma cells, while reduced TPA-induced levels of N-cadherin and vimentin on A375 cells. These data further support the evidence that GSPs function as a COX-2 inhibitor and have the ability to reverse EMT in melanoma cancer cells and thus lead to reduce the invasiveness of melanoma cells.

**Figure 6:** The effect of GSPs, TPA and celecoxib on the EMT biomarkers in melanoma cells. A375 cells were treated for 24 h and cell lysates were prepared for the analysis of N-cadherin, vimentin and desmoglein 2 using western blot analysis. Equal loading of proteins on the membranes were verified using β-actin antibody. Representative blots are shown from 3 independent experiments.

## Discussion

Melanoma cells can metastasize rapidly and that is the leading cause of death. According to a World Health Organization report, 48,000 melanoma-related deaths occur worldwide per year [21]. Treatment is more difficult if it has spread beyond skin and lymph nodes [22]. Therefore, innovative strategies are required to be developed for the prevention of the invasive or the migratory potential of melanoma cells. Many human cancers express elevated levels of COX-2 and enhanced biosynthesis of PGs. COX-2 overexpression and abundant production of PGs, and particularly PGE_2_, have been linked with tumor progression, invasion and metastasis [23]. Because of its important role in tumor invasion and metastasis, COX-2 is always a promising target for cancer therapy [8], [24]; therefore, the search and development of potential COX-2 as well as PGE_2_ inhibitors for the prevention or treatment of melanoma may prove to be an important and effective strategy.

RETRACTED

The significant findings in the present study are that the treatment of melanoma cells with GSPs inhibits cell migration in a dose-dependent manner, and that is associated with the inhibition of COX-2 expression and PGE_2_ production. The melanoma cells overexpress COX-2, and the inhibition of COX-2 by GSPs contributes to the inhibition of cell migration of these cells. This concept is supported by the evidence that treatment of the melanoma cells with celecoxib, a potent COX-2 inhibitor, resulted in a reduction in cell migration. Similar effects were also noted when the melanoma cancer cells, A375 and Hs294t, were transfected with COX-2 siRNA. It has been shown that TPA promotes COX-2 expression, and we found that treatment of melanoma cells with TPA enhances cell migration, and that this TPA-induced cell migration was blocked by the treatment of cells with GSPs. These observations support the evidence that inhibition of melanoma cell migration by GSPs requires the inhibition of COX-2 expression. It has been reported that COX-2 inhibitors can inhibit cell migration; however, they may also induce some form of toxicity. This possibility is not found in GSPs as these are dietary components and toxicity has not been observed in animal models [10], [11].

It is well known that PGE_2_ exerts its biologic functions by stimulating epithelial cell growth, invasion potential and cellular survival signals [25], [26]. Singh et al. [27] have shown that PGE_2_ treatment enhanced melanoma cell migration and that berberine, a phytochemical, inhibits PGE_2_-induced migration of melanoma cells. Punathil and Katiyar [28] have examined the effect of GSPs on non-small cell lung cancer cell migration, and found that GSPs inhibit the migration of these cells by targeting nitric oxide, guanylate cyclase and ERK1/2 pathways. As COX-2 is a downstream target of NF-κB pathway, we further checked the effect of GSPs on the basal levels of NF-κB in melanoma cells, and found that treatment of melanoma cells with GSPs results in inactivation of NF-κB pathway in a dose-dependent manner. GSPs down-regulate the levels of IKKα which is responsible for NF-κB activation. Treatment of melanoma cells with caffeic acid phenethyl ester, an inhibitor of NF-κB, resulted in an inhibitory effect on melanoma cell migration. These observations support the concept that the inhibitory effect of GSPs on melanoma cell migration is mediated through the downregulation of COX-2 and PGE_2_, which are the downstream targets of NF-κB. Our study also demonstrates the requirement of activated ERK1/2 in melanoma cancer cell migration. Our results show that inhibition of melanoma cell migration by GSPs is associated with the inhibition of ERK1/2 phosphorylation. The inhibition of MEK with UO126, a MEK inhibitor, blocked the migration capacity of melanoma cells which is similar to the action of GSPs. Treatment of A375 cells with TPA increased ERK1/2 phosphorylation and subsequently enhanced cell migration, while treatment of cells with celecoxib decreased ERK1/2 phosphorylation and subsequently decreased cell migration. These observations suggest a possible involvement of MAPK pathway (which is an upstream regulator of NF-κB) in inhibition of melanoma cell migration by GSPs.

RETRACTED

The transcription factor NF-κB regulates a wide spectrum of biological processes, including inflammation, cell proliferation and apoptosis. Additional roles of NF-κB in cancer biology, such as in tissue invasion, cell migration and metastasis, have been investigated recently. Importantly, NF-κB is involved in inflammation-induced cancer development, and has been identified as an important regulator of EMT in several cancer cell types [17]–[20]. EMT has been observed to play a major role in invasion and metastasis of epithelial tumors. EMT can render tumor cells migratory and invasive through the involvement of all stages, invasion, intravasation and extravasation [12]. During the process of EMT, cells can change from an epithelial to a mesenchymal state. They lose their characteristic epithelial traits and instead gain properties of mesenchymal cells. This process is primarily coordinated by the disappearance or loss of epithelial biomarkers such as E-cadherin and certain cytokeratins with the concomitant appearance or gain of mesenchymal markers such as vimentin, fibronection and N-cadherin, etc. In the present study, GSPs treatment of melanoma cells showed the suppression of mesenchymal biomarkers, such as vimentin, fibronectin and N-cadherin while restored the levels of epithelial biomarkers such as, E-cadherin, desmoglein 2, keratin-8 and -18, etc, in melanoma cells which suggest that GSPs have the ability to reverse the EMT process in melanoma cells and this may also be one of the possible mechanisms through which GSPs reduce the invasiveness of melanoma cells and that lead to inhibition of melanoma cell migration in our system.

RETRACTED

In summary, the results from this study have identified for the first time that GSPs inhibit the invasiveness of melanoma cells or inhibit the ability of melanoma cell migration and that involves: (i) the inhibitory effect of GSPs on endogenous COX-2 overexpression and successive down-regulation of PGE_2_ synthesis, (ii) the inhibitory effect of GSPs on the activation of NF-κB and the proteins of MAPK family, which are the upstream regulators of COX-2 and PGE_2_, and (iii) the reversal of EMT process. More detailed studies are needed to develop GSPs as a pharmacologically safe agent either alone or in combination with other anti-metastatic drugs for the treatment of metastatic melanoma in humans.
